# Effect Evaluation of Comfort Nursing Materials Assisted Nursing for Patients with Advanced Malignant Tumor

**DOI:** 10.1155/2022/4766252

**Published:** 2022-06-17

**Authors:** Mei Zhong, Lanying He, Min Chen, Zhongxiang Lu, Ruyu Li, Ling Li

**Affiliations:** Department of Intensive Care Medicine, Sun Yat-sen University Cancer Center, Guangzhou 510060, China

## Abstract

In order to explore the effect of comfort care on patients with advanced malignant tumors assisted by bioceramics, 82 patients with advanced malignant tumors admitted to a cancer hospital were selected as the research object control group: 26 males and 15 females and the observation group: 25 males and 16 females. The control group was given routine care, and the observation group was given comfort care on the basis of the control group. The quality of life (QLQ-C30 functional scale) and nursing satisfaction before and after nursing were compared between the two groups. The results of the study indicate that after care, the physical, role, emotional, cognitive, social, general health, and symptom scores of the observation group were significantly higher than those of the control group, the nursing satisfaction degree of the observation group was 97.56%, which was significantly higher than that of the control group of 82.93%, and the difference was statistically significant (*P* < 0.05). Comfortable care has a definite effect on the care of patients with advanced malignant tumors; it can improve the overall comfort and satisfaction of patients, effectively reduce adverse events, and improve the quality of life of patients.

## 1. Introduction

The body function of patients with advanced malignant tumors is reduced, there are more psychological problems, and the quality of life is significantly reduced; at the same time, the family members of the patients were also affected, and their psychological status was deviated. Therefore, effective interventions for patients and their families can help them alleviate bad psychology and improve the quality of life [1]. Comfort care was first proposed in the 1960s; studies believe that applying it to patients with advanced malignant tumors can play an important role, reflecting the value of his life. Advanced tumors mainly refer to the failure of cancer detection and treatment; once discovered, it is already at an advanced stage, which increases the difficulty of disease treatment. Pain is the most common subjective symptom in patients with advanced cancer, the probability of occurrence is as high as 70%; if timely and effective treatment is not available, it will reduce the quality of life of patients and increase the psychological pressure of patients [2, 3]. With the development of medical care reform, humanized nursing is applied to the treatment of advanced tumors, provides patients with personalized and creative care, solves the pain on the patient's body, and improves the patient's confidence in disease treatment [4].

Malignant tumors seriously affect the life and health of patients; at present, the clinical treatment of this malignant tumor is to first perform surgical treatment on the patient, complete removal of tumor tissue. And adjuvant chemotherapy and radiation therapy after surgery prevent the residue and metastasis of tumor cells, but the side effects of chemotherapy and radiotherapy are great [5]. For bone tumors, clinical treatment can also cause irreparable bone defects [6]. Therefore, the construction of selenium-doped potassium sodium niobate bioceramics is used to achieve bone defect filling and use the piezoelectric properties of the ceramic sheet and the released Se element to achieve an effective combination of electrotherapy and drug therapy to achieve the purpose of anticancer. For malignant tumors, construction of selenium-doped potassium sodium niobate ceramics, utilizing the photocatalytic performance of ceramic powder and the released Se element, can realize the effective combination of photodynamic therapy and drug therapy to achieve the purpose of anticancer. During the nursing of patients with advanced malignant tumors assisted by bioceramics, the principle should be to reduce the pain of patients and improve their quality of life. Traditional nursing methods cannot meet the care needs of patients. Th et al. investigated the prognosis of patients with stage I and stage II OSCC, especially the impact of biopsy and operation intervals; research has shown that preoperative interventions for patients with oral malignancies such as tooth extraction, incision, and curettage may be related to poor prognosis. Although biopsy is another preoperative intervention, its impact on the prognosis of patients with oral squamous cell carcinoma (OSCC) is unclear [7].

On the basis of this research, we observe the evaluation of the effect of comfortable nursing on the nursing of patients with advanced malignant tumors assisted by bioceramics. 82 patients with advanced malignant tumors were selected as the research objects. Using a random number table method, they were divided into the control group and observation group with 41 cases each. The control group was given routine care, and the observation group was given comfort care on the basis of the control group. The quality of life and nursing satisfaction of the two groups before and after nursing were compared. The physical, role, mood, cognition, social, general health, and symptom scores of the observation group were significantly higher than those of the control group. Using comfortable care on the basis of routine care can improve the quality of life of patients with advanced malignant tumors and improve nursing satisfaction.

## 2. Research Methods

### 2.1. General Information

82 patients with advanced malignant tumors admitted to a cancer hospital were selected as the research objects; all met the relevant standards in “Malignant Tumor Interventional Therapy” and signed an informed consent form. Using a random number table method, they were divided into the control group and observation group with 41 cases each. Control group: 26 males and 15 females; age 25-67 years old, average 45.7 ± 0.8 years old. The course of illness is 2-7 years, with an average of 4.9 ± 0.6 years; disease types: 14 cases of gastric cancer, 12 cases of esophageal cancer, 8 cases of liver cancer, 6 cases of cervical cancer, and 1 case of lung cancer. Observation group: 25 males and 16 females; age 25~68 years old, average 45.8 ± 0.9 years old. The course of the disease is 3 ~ 7 years, with an average of 4.8 ± 0.5 years; disease types: 13 cases of gastric cancer, 10 cases of esophageal cancer, 9 cases of liver cancer, 6 cases of cervical cancer, and 3 cases of lung cancer. There was no statistically significant difference between the two groups of general information (*P* > 0.05), and they were comparable.

### 2.2. Method

The control group was given routine care: ① provide patients with a quiet and comfortable ward environment; ensure fresh air, suitable temperature, and humidity; and disinfect the ward on time every day and dry the bedding to prevent pressure sores. ② In view of the digestive tract reactions that are prone to chemotherapy, 30 minutes before chemotherapy, give antiemetic drugs and sedatives as prescribed by the doctor. ③ For patients with mild pain, use cold compresses, physical therapy, and distraction to relieve pain. For patients with moderate to severe pain, use analgesics as directed by your doctor. The observation group was given comfort care on the basis of the control group: ① layout+ward environment according to patients' interests and hobbies, place green potted plants indoors and avoid noise during the nursing process and keep a quiet ward environment; ② pay attention to the psychological changes of patients, when communicating, think about the problem more from the perspective of the patient, pay attention to the use of communication skills, pour in your own emotions and establish a friendly nurse-patient relationship, gain the trust of patients, reduce their psychological pressure, and improve their confidence in treatment; ③ formulate an appropriate diet plan for the patient, focusing on digestible foods with high vitamin content, it is forbidden to eat too sweet and greasy food; instruct patients to drink plenty of water to promote the excretion of metabolites, and prevent constipation; ④ make appropriate exercise programs based on the patient's situation, such as walking, Tai Chi, jogging, etc., the first exercise time is 10~15 min, then gradually increased to 30 min, 2 ~ 3 times a week; ⑤ for patients with bone marrow suppression caused by chemotherapy, urge patients to pay attention to oral hygiene and maintain indoor ventilation, wear a mask when going out, and strictly restrict people entering and leaving the ward to prevent cross-infection.

### 2.3. Observation Indicators

The QLQ-C30 functional scale was used to assess the quality of life of the two groups of patients, including physical function, role function, emotional function, cognitive function, the seven dimensions of social function, general health, and symptoms, the full score is 100 points, the higher the score, the better the quality of life. A self-made questionnaire was used to calculate the nursing satisfaction of the two groups, the total score is 100 points, >90 points to satisfaction, 60 to 90 points to basic satisfaction, and <60 is divided into dissatisfaction: satisfaction = (satisfied + basic satisfaction) number of cases/total number of cases × 100%.

### 2.4. Potassium Sodium Niobate Bioceramics

Potassium sodium niobate piezoelectric ceramics have piezoelectric properties similar to those of natural bone tissue; the chemical elements contained in KNN are potassium, sodium, oxygen, and niobium; among them, potassium, sodium, and oxygen are all chemical elements required by the human body: niobium has also been proven to have a bone-promoting effect, and its biological safety has also been recognized. The biocompatibility of potassium sodium niobate piezoelectric ceramics has been confirmed, and its piezoelectric properties are used in antitumor research. At the same time, bioceramics have good photosensitivity; its photosensitivity can also be used for antitumor research. Under visible light, the conduction band and valence band of KNN photosensitive ceramics will generate photo-induced electrons and positively-charged photo-induced holes, respectively, cause a series of chemical redox reactions to occur in the substances in the solution and generate reactive oxygen species. Therefore, the use of bioceramics as a photocatalyst to achieve photodynamic therapy of cells has become a means of advanced malignant tumors.

### 2.5. Statistical Methods

Use SPSS 18.0 statistical software to process the data, and the measurement data is represented by ($\bar{x}\pm s$); *t*-test was used for comparison, *x*^2^ test was used for count data, and *P* < 0.05 was considered statistically significant.

## 3. Result Analysis

### 3.1. Comparison of Serum Tumor Standard Levels between the Two Groups

The serum levels of tumor markers such as CA-125, Cyfra21-1, and NSE in the observation group were significantly lower than those in the control group, and the difference was statistically significant (*P* < 0.05, Table 1).

### 3.2. Comparison of Quality of Life before and after Nursing between the Two Groups

Before care, two groups of physical function, role function, emotional function, cognitive function, social function, general health, there was no statistically significant difference in symptom scores (*P* > 0.05). After nursing, the observation group's body, role, emotion, cognition, the social, general health status, and symptom scores were significantly higher than those of the control group; the difference was statistically significant (*P* < 0.05), see Table 2.

### 3.3. Comparison of Nursing Satisfaction between the Two Groups

The nursing satisfaction degree of the observation group was 97.56%, which was significantly higher than that of the control group of 82.93%, and the difference was statistically significant (*P* < 0.05), see Table 3.

According to statistics, the treatment compliance of patients in the observation group after nursing was 84.8%, significantly higher than the 65.2% of the control group, and the treatment compliance of the two groups of patients after nursing was statistically different (*P* < 0.05). Comparing the pain relief of the two groups of patients, the pain relief effectiveness of the observation group was higher than that of the control group, and the difference was statistically different (*P* < 0.05), see Figure 1.

## 4. Discussion

Comfortable care is the most pleasant state for patients to obtain physical, psychological, and social functions during treatment, in order to achieve the above goals, an effective, holistic, creative, and personalized nursing model should be established in clinic and meet the needs of patients to the greatest extent and from multiple angles [8, 9]. For patients with malignant tumors receiving chemotherapy and radiotherapy, comfortable care mode mainly includes basic comfort care, pain care, clinical symptom care, psychosocial care, and adverse reaction care, it can significantly improve the clinical treatment effect, improve the quality of life of patients, and relieve symptoms; it can also reduce the adverse reactions of radiotherapy and chemotherapy and improve patient tolerance, ensuring the smooth progress of clinical treatment [10–12].

At present, with the continuous increase in the incidence of various malignant tumors, cancer pain has become a problem that medical staff cannot ignore. Pain not only affects the patient's body but also puts a huge shackle on the patient's psychology. This requires that the implementation of pain care for patients should start from the “physical, psychological, and social spirit” at the same time to carry out the “trinity” holistic care; this is a challenge to the current role change of medical staff and the level of care [13]. In order to effectively improve the nursing staff's pain nursing service skills, the hospital should regularly arrange nursing staff to participate in pain management lectures, strengthen the pain management awareness of medical staff by organizing various channels such as “teaching, further training, and going out to study” and accurately grasp the assessment method of cancer pain; on the basis of continuous and accurate pain assessment, we strictly abide by the three-step analgesic principle formulated by the WHO and implement corresponding pain care measures [14]. For patients with advanced malignant tumors, comprehensive nursing intervention can play a good role in pain control; nursing staff should not only pay attention to the patient's symptoms and pain, through correct assessment and scientific pain management, at the same time, patients should be given a clean and quiet ward, by strengthening psychological counseling to meet the needs of patients as much as possible, so that patients can maintain a positive attitude to face the disease, so as to effectively alleviate the pain of patients and improve their compliance with treatment, in order to ensure the quality of life in the late stage, so that patients can spend this time comfortably and peacefully [15–17].

Patients with advanced malignant tumors have a short survival time, affected by the disease, patients and their families are under great psychological pressure, and most patients have severe cancer pain, and their quality of life is significantly reduced. We apply comfort care interventions to the treatment of patients with malignant tumors; the results showed that the general nursing group performed basic general nursing, and the comfort care group gives comfort care [18]. The results show that the satisfaction of nursing care for advanced malignant tumors in the comfort nursing group was higher than that in the general nursing group, *P* < 0.05. Before the intervention, the physical health, mental health, social function, and overall quality of life of the two groups were similar, *P* > 0.05. After the intervention, the physical health, mental health, social function, and overall quality of life of the comfortable nursing group were better than those of the ordinary nursing group, *P* < 0.05. The comfort care group nursing operation comfort, speech comfort, and the comfort of the ward environment are 97.40 ± 4.57 points, 96.61 ± 2.51 points, and 97.40 ± 2.87, which were higher than the score of 85.51 ± 2.62, 85.62 ± 1.88, and 89.51 ± 1.21 of the general nursing group, *P* < 0.05. The incidence of adverse nursing events in the comfort care group was 2.50% lower than 20.00% in the general care group, *P* < 0.05.

For patients with advanced malignant tumors, chemotherapy is often given clinically; although it can get a certain effect, it is easy to cause vomiting, nausea, and other adverse reactions, coupled with the particularity of the disease, affecting patient comfort. Routine care cannot meet the needs of patients for care [19–21]. Comfort care is a new type of care model that follows the patient-centered concept and meets the psychological and physical needs of patients; the patient can feel the respect and care of the nursing staff, thereby improving the comfort of the patient. The results of this study show that the observation group's body, role, emotion, cognition, society, general health status, symptom score, and nursing satisfaction were significantly higher than those of the control group. This is because it strengthens communication with patients during comfort care and comprehensively evaluates the psychological condition of patients, choosing effective measures to guide can not only meet the physical and psychological needs of patients but also allows patients to feel the care from society and family during their hospitalization, so as to improve its treatment compliance and ensure the treatment and nursing effect [22–24]. At the same time, preaching disease knowledge to patients and guiding them to perform aerobic exercises can improve the patient's health knowledge mastery, self-care awareness, and autonomy. Combining the patient's condition to formulate a scientific and reasonable diet plan can increase the body's nutrition and improve the quality of life [25].

## 5. Conclusion

In summary, the effect of comfort care on the nursing of patients with advanced malignant tumors assisted by bioceramics is definite; it can improve the overall comfort and satisfaction of patients. It can not only reduce the pain and anxiety of patients but also enhance their nursing satisfaction, effectively reduce adverse events, and improve the quality of life of patients.

## Figures and Tables

**Figure 1:** Comparison of pain relief between the two groups of patients after nursing.

**Table 1:** Comparison of serum tumor marker levels between the two groups of patients ($\bar{x}\pm s$).

Tumor markers	Observation group (*n* = 913)		Control group (*n* = 710)	
	Before care	After care	Before care	After care
CA-125	87.91 ± 4.54	43.66 ± 2.12	29.11 ± 3.56	67.15 ± 2.83
Cyfra21-1	5.92 ± 0.48	2.05 ± 0.21	6.26 ± 0.53	3.87 ± 0.24
NSE	37.92 ± 2.05	17.41 ± 1.93	38.46 ± 2.41	23.63 ± 1.88

**Table 2:** Comparison of quality of life between the two groups before and after nursing.

Project	Observation group (*n* = 41)		Control group (*n* = 41)	
	Before care	After care	Before care	After care
Physical function	32.24 ± 5.10	54.20 ± 6.18^∗^^#^	32.20 ± 5.11	45.28 ± 4.62^#^
Role function	39.51 ± 4.57	53.61 ± 6.43^∗#^	39.47 ± 4.41	44.65 ± 4.31^#^
Emotional function	40.54 ± 4.77	52.50 ± 5.38^∗^^#^	40.62 ± 4.83	46.02 ± 4.91^#^
Cognitive function	40.10 ± 4.21	55.22 ± 5.64^∗^^#^	40.01 ± 4.16	47.60 ± 4.62^#^
Social function	38.84 ± 3.45	54.44 ± 5.62^∗^^#^	38.78 ± 3.38	48.05 ± 4.50^#^
Symptom	41.10 ± 6.13	52.80 ± 5.70^∗^^#^	41.15 ± 6.02	45.12 ± 5.68^#^
General health	39.24 ± 6.01	59.20 ± 5.73^∗^^#^	39.17 ± 5.95	47.21 ± 5.03^#^

Note: compared with the control group, ^∗^*P* < 0.05; compared with before nursing, ^#^*P* < 0.05.

**Table 3:** Comparison of nursing satisfaction between the two groups (*n* (%)).

Group	Satisfy	Basically satisfied	Dissatisfied	Satisfaction
Observation group (*n* = 41)	17 (42.8)	21 (53.65)	1 (2.43)	39 (97.55)
Control group (*n* = 41)	13 (34.14)	19 (48.76)	6 (17.06)	343 (82.92)
*x* ^2^ value				3.462
*P* value				0.025

## Data Availability

The data used to support the findings of this study are available from the corresponding author upon request.
